The article "5-HT induces PPAR γ reduction and proliferation of pulmonary artery smooth muscle cells via modulating GSK-3β/β-catenin pathway" was published in 2017. Journal: Oncotarget.

# 5-HT induces PPAR γ reduction and proliferation of pulmonary artery smooth muscle cells via modulating GSK-3β/β-catenin pathway

**DOI:** 10.18632/oncotarget.20582

**Published:** 2017-08-24

**Authors:** Rui Ke, Xinming Xie, Shaojun Li, Yilin Pan, Jian Wang, Xin Yan, Weijin Zang, Li Gao, Manxiang Li

**Affiliations:** ^1^ Department of Respiratory Medicine, the First Affiliated Hospital of Xi'an Jiaotong University, Xi'an, Shaanxi 710061, China; ^2^ Department of Pharmacology, Xi'an Jiaotong University Health Science Center, Xi'an, Shaanxi 710061, China; ^3^ Division of Allergy and Clinical Immunology, Department of Medicine, The Johns Hopkins University School of Medicine, Baltimore, MD 21224, USA

**Keywords:** PPAR γ, β-catenin, GSK-3β, PASMCs, proliferation

## Abstract

Studies have shown that peroxisome proliferator-activated receptor γ (PPAR γ) is down-regulated in pulmonary vascular lesions of patients with pulmonary hypertension (PH) and animal models of PH. Yet, the detailed molecular mechanisms underlying this alteration are not fully defined; the aim of this study is to address this issue. 5-HT dose- and time-dependently reduced PPAR γ expression and promoted pulmonary artery smooth muscle cells (PASMCs) proliferation; this was accompanied with the phosphorylation of Akt, inactivation of GSK-3β and up-regulation of β-catenin. Importantly, pre-treatment of cells with PI3K inhibitor (Ly294002) or prior silencing of β-catenin with siRNA blocked 5-HT-induced PPAR γ reduction and PASMCs proliferation. In addition, inactivation or lack of GSK-3β or inhibition of proteasome function up-regulated β-catenin protein without affecting its mRNA level and reduced PPAR γ protein expression. Taken together, our study indicates that 5-HT suppresses PPAR γ expression and stimulates PASMCs proliferation by modulating GSK-3β/β-catenin axis, and suggests that targeting this pathway might have potential value in the management of PH.

## INTRODUCTION

Pulmonary hypertension (PH) is a common clinical syndrome characterized by sustained elevation of pulmonary vascular resistance and increased pulmonary arterial pressure, leading to right heart failure and ultimately death [1]. All types of PH share similar pathogenesis including vasoconstriction, pulmonary vascular remodeling and thrombosis in situ [2]. Pulmonary vascular remodeling characterized by thickening of all layers of vascular wall is a hallmark of PH [3], and pulmonary arterial smooth muscle cells (PASMCs) proliferation is critical in this process [4]. Therefore, exploring the molecular mechanisms responsible for PASMCs proliferation and searching for new targets are important in the management of PH.

Peroxisome proliferator-activated receptor γ (PPAR γ) is a member of the PPAR nuclear hormone receptor superfamily. Besides its metabolic actions [5], emerging evidences have demonstrated that PPAR γ regulates diverse cellular processes including cell proliferation, apoptosis, differentiation and migration [6, 7]. It has been found that PPAR γ is expressed in most of tissues including pulmonary system and its expression is down-regulated in pulmonary vasculature of patients with PH [8]. Further studies have demonstrated that genetic deletion of PPAR γ in mice pulmonary vascular SMCs is sufficient to causes spontaneous PH [9], while activation of PPAR γ strongly attenuates PASMCs proliferation and inhibits the development of PH [10–12]. PPAR γ insufficiency has been considered to be a crucial factor for the development of PH by stimulating PASMCs proliferation and therefore vascular remodeling. However, the exact mechanisms underlying down-regulation of PPAR γ in PASMCs of PH are still largely unknown.

The Wnt/β-catenin signaling pathway controls many biological processes including cell proliferation, apoptosis and differentiation [13]. β-catenin is a key effector in this pathway. The absence of Wnts facilitates the phosphorylation of β-catenin protein by glycogen synthase kinase-3β (GSK-3β), leading to β-catenin ubiquitination and degradation, whereas Wnts induces the phosphorylation and inactivation of GSK-3β and subsequent stabilization of β-catenin protein. The resulting increased free β-catenin then shift into the nucleus regulating expression patterns of target genes [14]. Studies have shown that accumulated β-catenin translocate to the nucleus and suppress PPAR γ expression in a variety of tumor cells and non-pulmonary arterial smooth muscle cells [15–18]. Therefore, it is interesting to examine whether activation of β-catenin signaling suppresses PPAR γ expression in PASMCs and implicates in PASMCs proliferation. To clarify this, primary cultured PASMCs were stimulated with 5-HT, a potent mitogen that has been shown to be associated with the development of PH. The phosphorylation of GSK-3β and the expression of β-catenin and PPAR γ were determined, and the molecular mechanisms underlying these changes were further investigated.

## RESULTS

### 5-HT stimulates PASMCs proliferation

To examine the effect of 5-HT on PASMCs proliferation, dose-response and time-course of 5-HT on cell proliferation were investigated. Cell proliferation was determined by BrdU incorporation assay. As shown in Figure 1A, 5-HT dose-dependently stimulated PASMCs proliferation, 1 μM 5-HT triggered a 1.59-fold increase in BrdU incorporation at 24 h compared with control (*P* < 0.01). Figure 1B demonstrates that 5-HT stimulated PASMCs proliferation in a time-dependent manner, 1 μM 5-HT caused a 1.75-fold increase in BrdU incorporation over control at the time of 72 h (*P* < 0.01), indicating that 5-HT effectively stimulates PASMCs proliferation.

**Figure 1:** 5-HT stimulates PASMCs proliferation **(A)** PASMCs were stimulated with different concentration of 5-HT ranging from 0 to 10000 nM for 24 h, the rate of BrdU incorporation in cells was determined using BrdU ELISA assay Kit (n = 4 each group). **(B)** Cells were exposed to 1 μM 5-HT for the indicated times, BrdU incorporation in cells was measured (n = 4 each group). *P < 0.05 versus control; **P < 0.01 versus control.

### 5-HT reduces PPAR γ expression in PASMCs

To clarify whether 5-HT reduces PPAR γ expression in PASMCs, cells were treated with different concentration of 5-HT at different time point and the protein level of PPAR γ was determined using Western blotting. As indicated in Figure 2A, 5-HT dose-dependently down-regulated PPAR γ expression in PASMCs at 24 h, 1 μM 5-HT reduced PPAR γ protein level to 0.51-fold compared with control (*P* < 0.01). Figure 2B shows the time course of 1 μM 5-HT regulation of PPAR γ protein level, which dropped to 0.41-fold compared with control at the time of 72 h (*P* < 0.01). These results suggest that 5-HT suppresses PPAR γ expression in PASMCs.

**Figure 2:** 5-HT suppresses PPAR γ expression in PASMCs **(A)** PASMCs were treated with different concentration of 5-HT ranging from 0 to 10000 nM for 24 h, protein level of PPAR γ was determined using immunoblotting, GAPDH served as loading control (n = 4 each group). **(B)** Cells were incubated with 1 μM 5-HT for the indicated times, protein level of PPAR γ was assayed. GAPDH served as loading control (n = 4 each group). *P < 0.05 versus control; **P < 0.01 versus control.

### 5-HT inactivates GSK-3β, up-regulates β-catenin and reduces PPAR γ via PI3K/Akt pathway

It has been shown that activation of PI3K/Akt signaling pathway phosphorylates GSK-3β at Ser 9 resulting in inactivation of GSK-3β and subsequent inhibition of β-catenin degradation in several types of non-pulmonary arterial smooth muscle cells [19, 20]. To examine whether this mechanism also works in PASMCs and mediates 5-HT-induced PPAR γ reduction, PASMCs were prior incubated with Ly294002 (25 μM, a selective PI3K inhibitor) for 30 min and followed stimulation with 1 μM 5-HT, the phosphorylation of Akt and GSK-3β and the protein levels of β-catenin and PPAR γ were determined using Western blotting. Figure 3A and 3B show that 1 μM 5-HT stimulation for 5 min notably increased the phosphorylation levels of Akt and GSK-3β in PASMCs, while pre-treatment of cells with Ly294002 suppressed 5-HT-induced phosphorylation of Akt and GSK-3β. Phosphorylation of Akt declined from 2.06-fold increase over control in 5-HT-treated cells to 0.91-fold over control in Ly294002 and 5-HT-treated cells (*P* < 0.01), and phosphorylation of GSK-3β dropped from 1.99-fold over control in 5-HT-treated cells to 1.09-fold over control in Ly294002 and 5-HT-treated cells (*P* < 0.01). Figure 3C indicates that 1 μM 5-HT stimulation for 24 h resulted in a 1.98-fold increase in β-catenin protein level compared with control (*P* < 0.01), while pre-incubation of cells with Ly294002 reduced β-catenin protein level to 1.23-fold over control in response to 5-HT (*P* < 0.01 versus 5-HT-treated cells). Furthermore, the presence of Ly294002 dramatically blocked 5-HT-induced PPAR γ protein reduction, which increased from 0.5-fold over control in 5-HT-treated cells to 0.87-fold over control in Ly294002 and 5-HT co-treated cells (Figure 3D, *P* < 0.01). These results suggest that 5-HT inactivates GSK-3β, up-regulates β-catenin and reduces PPAR γ expression via PI3K/Akt pathway.

**Figure 3:** 5-HT inactivates GSK-3β, up-regulates β-catenin and reduces PPAR γ by PI3K/Akt pathway PASMCs were pre-treated with 25 μM Ly294002 for 30 min and followed stimulation with 1 μM 5-HT for 5 min, the phosphorylation of Akt **(A)** and GSK-3β **(B)** were determined using immunoblotting. Representative western blot and quantification of bands are shown (n = 4 each group). PASMCs were pre-incubated with 25 μM Ly294002 for 30 min before stimulation with 1 μM 5-HT for 24 h, the protein levels of β-catenin **(C)** and PPAR γ **(D)** were examined by immunoblotting. GAPDH served as loading control (n = 4 each group). *P < 0.01 versus control; #*P* < 0.01 versus 5-HT-treated cells.

### GSK-3β insufficiency or inhibition of proteasome function up-regulates β-catenin and reduces PPAR γ in PASMCs

Studies have shown that β-catenin stability and consequent its overall amount in cell is finely regulated by GSK-3β and proteasome system in mammalian cells [21, 22]. To investigate whether the level of β-catenin was also regulated by GSK-3β and proteasome function in PASMCs, inactivation/depletion of GSK-3β or proteasome inhibitor MG132 was applied in the study. Figure 4A indicates that transfection of GSK-3β specific siRNA for 48 h in PASMCs reduced GSK-3β protein level to 21% of control (*P* < 0.01), while non-targeting siRNA did not affect GSK-3β protein level. Figure 4B shows that β-catenin mRNA level did not change in PASMCs exposed to 1 μM 5-HT for 24 h or transfected with GSK-3β siRNA for 48 h or incubated with proteasome inhibitor MG132 (10 μM) for 24 h compared with control. However, these cells exhibited a significant increase in β-catenin protein level, which raised to 1.91-fold, 1.95-fold and 1.84-fold over control, respectively (Figure 4C, *P* < 0.01).

**Figure 4:** GSK-3β insufficiency or inhibition of proteasome activity up-regulates β-catenin and reduces PPAR γ **(A)** PASMCs were transfected with GSK-3β sequence-specific siRNA and non-targeting siRNA for 48 h. Equal amount of protein was loaded and probed with antibodies against GSK-3β and GAPDH (loading control) (n = 4 each group). **(B-D)** PASMCs were incubated with 1 μM 5-HT for 24 h or transfected with GSK-3β siRNA for 48 h or treated with 10 μM MG132 for 24 h, the mRNA level of β-catenin (B) was examined by qRT-PCR, GAPDH served as an internal control (n=4 each group); protein levels of β-catenin (C) and PPAR γ (D) were determined using immunoblotting, GAPDH served as an internal control (n=4 each group) *P < 0.05 versus control; **P < 0.01 versus control.

To examine whether inactivation/loss of GSK-3β or suppression of proteasome function results in PPAR γ reduction in PASMCs, cells were incubated with 1 μM 5-HT for 24 h or transfected with GSK-3β siRNA for 48 h or treated with 10 μM MG132 for 24 h, the protein level of PPAR γ was determined using Western blotting. Figure 4D shows that inactivation or depletion of GSK-3β decreased PPAR γ protein level in PASMCs, which declined to 0.51-fold over control in 5-HT-stimulated cells and to 0.58-fold over control in GSK-3β siRNA transfected cells, respectively (*P* < 0.01). Suppression of proteasome function by MG132 also reduced PPAR γ protein level, which decreased to 0.67-fold compared with control (*P* < 0.05). Together, these results suggest that inhibition of GSK-3β or proteasome function leads to accumulation of β-catenin protein and reduction of PPAR γ protein.

### Up-regulation of β-catenin mediates 5-HT-induced PPAR γ reduction in PASMCs

To verify whether up-regulation of β-catenin specifically mediated 5-HT-induced PPAR γ reduction in PASMCs, cells were first transfected with β-catenin sequence specific siRNA for 24 h and then stimulated with 1 μM 5-HT for an additional 24 h, PPAR γ protein level was measured using immunoblotting. As shown in Figure 5A, β-catenin specific siRNA transfection for 48 h reduced β-catenin protein level to 22% of control (*P* < 0.01), while non-targeting siRNA did not affect β-catenin protein level. Figure 5B indicates that 1 μM 5-HT dramatically reduced PPAR γ protein level (*P* < 0.01 versus control), while loss of β-catenin reversed 5-HT-induced PPAR γ reduction, which increased from 0.50-fold over control in 5-HT-treated cells to 0.89-fold over control in 5-HT-treated cells with prior knockdown of β-catenin (*P* < 0.01). These results suggest that up-regulation of β-catenin particularly mediates 5-HT inhibition of PPAR γ expression in PASMCs.

**Figure 5:** Up-regulation of β-catenin mediates 5-HT-induced PPAR γ reduction **(A)** PASMCs were transfected with β-catenin sequence-specific siRNA and non-targeting siRNA for 48 h. Equal amount of protein was loaded and probed with antibodies against β-catenin and GAPDH (loading control) (n = 4 each group). **(B)** Cells were prior transfected with non-targeting siRNA or β-catenin specific siRNA for 24 h before stimulation with 1 μM 5-HT for an additional 24 h. Protein level of PPAR γ was determined using immunoblotting, GAPDH served as loading control (n = 4 each group). *P < 0.01 versus control; #*P* < 0.01 versus 5-HT-treated cells.

### Up-regulation of β-catenin and subsequent PPAR γ reduction mediates 5-HT-stimulated PASMCs proliferation

To clarify whether accumulation of β-catenin by GSK-3β inactivation and subsequent PPAR γ reduction are involved in 5-HT-induced PASMCs proliferation, cells were pre-incubated with 25 μM Ly294002 for 30 min or prior transfected with β-catenin siRNA for 24 h or pre-treated with 10 μM pioglitazone for 30 min and then stimulated with 1 μM 5-HT for an additional 24 h, the proliferation of cells was determined by BrdU incorporation assay. As shown in Figure 6, pre-incubation of cells with Ly294002 or prior silencing of β-catenin with siRNA abolished 5-HT-induced PASMCs proliferation as indicated by BrdU incorporation rate, which was reduced from 1.59-fold over control in 5-HT-treated cells to 1.06-fold over control in Ly294002 and 5-HT-treated cells and to 1.10 fold over control in β-catenin siRNA transfected and 5-HT-treated cells, respectively (*P* < 0.01). In addition, prior treatment of PASMCs with pioglitazone also suppressed 5-HT-induced cell proliferation, BrdU incorporation rate declined from a 1.59-fold increase over control in 5-HT-treated cells to a 1.16-fold increase over control in pioglitazone and 5-HT co-treated cells (*P* < 0.01). These results suggest that post-transcriptional up-regulation of β-catenin and subsequent PPAR γ reduction mediates 5-HT-induced PASMCs proliferation.

**Figure 6:** Up-regulation of β-catenin and subsequent PPAR γ reduction mediates 5-HT-stimulated PASMCs proliferation PASMCs were pre-incubated with 25 μM Ly294002 for 30 min or prior transfected with β-catenin siRNA for 24 h or pre-treated with 10 μM pioglitazone for 30 min and then stimulated with 1 μM 5-HT for an additional 24 h, cells proliferation was determined by BrdU incorporation assay. (n = 4 each group). *P < 0.01 versus control; #*P* < 0.01 versus 5-HT-treated cells.

## DISCUSSION

In this study, we have shown that 5-HT causes the reduction of PPAR γ expression in primary cultured PASMCs, this effect is coupled to the phosphorylation of Akt and inactivation of GSK-3β and subsequent post-transcriptional up-regulation of β-catenin, which further suppresses the expression of PPAR γ and leads to PASMCs proliferation. Our study provides novel molecular insight for 5-HT down-regulation of PPAR γ and stimulation of PASMCs proliferation.

Insufficiency of PPAR γ has been shown to be associated with the development of a variety of cancer and other human diseases, while activation of PPAR γ suppresses both tumor and normal cell proliferation [23–25]. Recent studies have further indicated that PPAR γ expression is reduced in pulmonary vascular lesions of PH patients and several PH experimental models [8, 26, 27]. Activation of PPAR γ by several chemical compounds or signaling pathways attenuates PH by inhibiting PASMCs proliferation and therefore pulmonary vascular remodeling [10–12, 28, 29]. Studies have shown that PPAR γ exerts anti-proliferative effects on PASMCs through multiple mechanisms, such as inhibition of store-operated calcium entry, induction of heme oxygenase (HO)-1, stabilization of cyclin-dependent kinase inhibitors, prevention of the increase of MicroRNA-21 and decrease of its target genes [10, 30–32]. These studies highlight the importance of PPAR γ as a central anti-proliferative regulator of vascular homeostasis in PH. However, the detailed molecular mechanisms underlying PPAR γ reduction occurred in PH remain largely unclear.

Wnt/β-catenin pathway plays an essential role in cell fate decision [13]. Numerous studies have shown that Wnt/β-catenin signaling is implicated in a variety of human disorders, including cancer, diabetes, osteoarthritis and cardiovascular diseases [33–35]. Recent studies have found that activation of this pathway is associated with abnormal PASMCs proliferation and vascular remodeling in PH [36, 37]. β-catenin is a crucial effect molecule in Wnt/β-catenin signaling [13]. Stabilization and accumulation of intracellular β-catenin result in its nuclear translocation, which impacts expression patterns of target genes [14]. Accumulation of β-catenin has been found to translocate to the nucleus and suppress PPAR γ expression in several types of non-pulmonary arterial smooth muscle cells [15–18]. Our present study shows that the elevation of β-catenin protein was accompanied with the reduction of PPAR γ and PASMCs proliferation in response to 5-HT. Silencing of β-catenin with siRNA abolished 5-HT-induced PPAR γ reduction and therefore suppressed PASMCs proliferation. These results suggest that PPAR γ is a specific target of β-catenin pathway in regulation of PASMCs proliferation.

GSK-3β is a serine/threonine protein kinase that regulates cell proliferation and apoptosis through multiple intracellular signaling pathways [38, 39]. GSK-3β negatively modulates Wnt/β-catenin signaling in mammalian cells [40, 41], which is constitutively active in resting cells [42] and is inactivated by several upstream protein kinases such as Akt, protein kinase A (PKA), p90 ribosomal S6 kinase (p90Rsk), p70 ribosomal S6 kinase (p70S6K) in response to extracellular stimulations [39, 43]. Studies have indicated that activation of PI3K/Akt signaling phosphorylates GSK-3β at Ser 9 resulting in inactivation of GSK-3β and subsequently inhibiting the degradation of β-catenin in non-vascular smooth muscle cell types [19, 20]. In this study, we found that 5-HT also phosphorylated GSK-3β at Ser9 and induced β-catenin up-regulation and PPAR γ reduction through PI3K/Akt pathway in PASMCs. We further showed that inactivation/deletion of GSK-3β or inhibition of proteasome function increased the protein level of β-catenin without affecting its mRNA level and reduced PPAR γ protein expression in PASMCs. Inhibition of PI3K/Akt cascade or knockdown of β-catenin reversed 5-HT-induced PPAR γ down-regulation and PASMCs proliferation, while activation of PPAR γ by pioglitazone suppressed 5-HT-induced cells proliferation. These results suggest that 5-HT inactivates GSK-3β through PI3K/Akt pathway and then post-transcriptionally up-regulates β-catenin, which in turn suppresses the expression of PPAR γ and leads to PASMCs proliferation.

## MATERIALS AND METHODS

### Cell preparation and culture

Primary PASMCs from main pulmonary arteries were prepared from Sprague-Dawley rats (70–80 g) according to the method reported by Wu et al [44]. All animal care and experiments were performed in accordance with the Guide for the Care and Use of Laboratory Animals of Xi'an Jiaotong University Animal Experiment Center. All protocols used in this study were approved by the Laboratory Animal Care Committee of Xi'an Jiaotong University. Briefly, pulmonary arteries were rapidly isolated from sacrificed rats, washed in phosphate buffered saline (PBS, 4°C), and dipped into Dulbecco's Modified Eagle Medium (DMEM, Gibco, Grand Isle, NY, USA) containing 10% fetal bovine serum (FBS, Sijiqing, HangZhou, China), 100 U/mL penicillin, and 100 μg/mL streptomycin. A thin layer of the adventitia was gently stripped off with a forceps and the endothelium was carefully removed by scratching the intima surface with an elbow tweezers. The remaining smooth muscle was cut into 1-mm tissue blocks and placed into a culture flask and then incubated in a 37°C, 5% CO_2_ humidified incubator. PASMCs were passaged using 0.25% trypsin (Invitrogen, Carlsbad, CA, USA) till reaching 80% confluence. All experiments were performed using cells between passages 3 and 6. The purity of PASMCs was determined by immunostaining with α-smooth muscle actin (α-SMA, Sigma, St Louis, MO, USA) as described previously. Fluorescence microscope images indicated that cells contained more than 90% of PASMCs (data not shown here). Before each experiment, cells were incubated in 1% FBS-DMEM overnight to minimize serum-induced effects. 5-HT (Sigma) was used to stimulate cell proliferation. Ly294002 (Sigma) was applied to inhibit PI3K activity. MG132 (Selleck Chemicals, Houston, TX, USA) was used as a selective proteasome inhibitor. Pioglitazone (Cayman Chemical Co., Ann Arbor, MI, USA) was used to stimulate PPAR γ activation.

### siRNA transfection

To silence the expression of GSK-3β or β-catenin protein, PASMCs were transfected with sequence-specific or non-targeting control siRNA (GenePharm, Shanghai, China) using Lipofectamine™ 2000 reagent (Invitrogen) according to the manufacture's protocols. Briefly, PASMCs were seeded into 6-well plates and cultured till reaching 30-40% confluence; 100 nM siRNA and 5 μL Lipofectamine were diluted in 250 μL DMEM, separately, and incubated for 5 min at room temperature. Diluted siRNA was mixed with diluted Lipofectamine and incubated at room temperature for 20 min. Then, the complex of siRNA and Lipofectamine was added into cells and cells were cultured for 48 h at 37°C, 5% CO_2_ in a humidified incubator. Effects of siRNA transfection were analyzed using immunoblotting.

### BrdU incorporation assay

To determine PASMCs proliferation, the rate of BrdU incorporation was examined using BrdU ELISA Kit (Maibio, Shanghai, China) following the established protocol. PASMCs were seeded on 96-well plates at 5×10^3^ cells per well, allowing to adhere for at least 24 h, and serum starved overnight (1% FBS in DMEM) before the start of experiments. After different treatments, BrdU labeling reagent was added to the wells and incubated for 2 h at 37°C. Cells were then denatured with FixDenat solution for 30 min, and incubated with anti-BrdU mAbs conjugated to peroxidase for 90 min at room temperature. After incubation, antibody conjugate was removed and substrate solution was added for reaction for 10 min. Finally, the reaction product was quantified by measuring the absorbance at 370 nm using a microplate reader (Bio-Rad, Richmond, CA, USA). The blank corresponded to 100 μL of culture medium with or without BrdU.

### Real-time PCR

Total RNA was extracted from primary cultured PASMCs with Trizol (Invitrogen) following the manufacturer's instructions. Expression of β-catenin and glyceraldehyde-3-phosphate dehydrogenase (GAPDH) mRNA was determined using Real-time PCR. Complementary DNA (cDNA) was synthesized with the cDNA Synthesis Kit (Takara, Tokyo, Japan). Real-time PCR was carried out on an IQ™5 Real-time PCR Detection System (Bio-Rad) using SYBR premix Ex Taq II (Takara) as fluorescent dye. The primers for β-catenin (Sangon Biotech, Shanghai, China) were: forward 5′-CCACGACTAGTTCAGCTGCTTGTAC-3′ and reverse 5′-ACTGCACAAACAGTGGAATGGTATT-3′. Primers for GAPDH (Sangon Biotech) were: forward 5′-GCTGAGTATGTCGTGGAGT-3′ and reverse 5′-GTTCACACCCATCACAAAC-3′. The PCR amplification was performed at 95°C for 1 min, followed by 40 cycles of 95°C for 5 s, 60°C for 20 s and 72°C for 30 s. Expression level of β-catenin was presented as fold increase over controls after normalization with GAPDH.

### Immunoblotting

The cultured cells were washed twice with ice-cold PBS and then lysed in RIPA lysis buffer containing 50 mM Tris/HCl (pH 7.4), 1% Nonidet P-40, 0.1% sodium dodecyl sulfate (SDS), 150 mM NaCl, 0.5% sodium deoxycholate, 1 mM EDTA, 1 mM phenylmethanesulfonyl fluoride, 1 mM Na3VO4, 1 mM NaF and proteinase inhibitors. Lysates were centrifuged at 13,000 rpm at 4°C for 15 min, and the supernatant was collected as sample protein. Protein was separated on SDS-PAGE gel and transferred to a nitrocellulose (NC, Bio-Rad) membrane via semidry transfer. The NC membrane was then blocked with 5% (w/v) nonfat dry milk in PBS containing 0.1% (v/v) Tween-20. Polyclonal or monoclonal antibodies against phosphor-Akt, total-Akt, phosphor-GSK-3β, total-GSK-3β, β-catenin (Cell Signaling Technology, Beverly, MA, USA, 1:1000 dilution), PPAR γ (Proteintech Group, Chicago, IL, USA, 1:500 dilution) as well as GAPDH (Sigma, 1:2000 dilution) were used according to the manufacturer's protocols. Horseradish peroxidase-conjugated goat anti-rabbit IgG was used as the secondary antibodies (Sigma, 1:5000 dilution). Reactions were visualized with SuperSignal West Pico Chemiluminescent Substrate (Pierce Biotechnology, Rockford, IL, USA) and then exposed to the autoradiographic film. Signaling was quantified from scanned films using Quality One software (Bio-Rad). Band quantification of aimed proteins was standardized by GAPDH or related total protein.

### Statistics

Statistical analysis was carried out using the SPSS 13.0 software. All values are presented as mean ± standard deviation (S.D.). Data were analyzed using one-way analysis of variance (ANOVA) with Tukey post hoc test. Probability values of P < 0.05 were considered to represent a statistically significant between groups.

## Abbreviations

GSK-3β: glycogen synthase kinase-3β
PI3K: phosphatidylinositol 3-kinase
PH: pulmonary hypertension
PASMCs: pulmonary artery smooth muscle cells
PPAR γ: peroxisome proliferator-activated receptor γ
5-HT: 5-hydroxytryptamine.

## References

[1] Galiè N, Humbert M, Vachiery JL, Gibbs S, Lang I, Torbicki A, Simonneau G, Peacock A, Vonk Noordegraaf A, Beghetti M, Ghofrani A, Gomez Sanchez MA, Hansmann G (2016). 2015 ESC/ERS Guidelines for the diagnosis and treatment of pulmonary hypertension. Eur Heart J.

[2] Schermuly RT, Ghofrani HA, Wilkins MR, Grimminger F (2011). Mechanisms of disease: pulmonary arterial hypertension. Nat Rev Cardiol.

[3] Vaillancourt M, Ruffenach G, Meloche J, Bonnet S (2015). Adaptation and remodelling of the pulmonary circulation in pulmonary hypertension. Can J Cardiol.

[4] Tajsic T, Morrell NW (2011). Smooth muscle cell hypertrophy, proliferation, migration and apoptosis in pulmonary hypertension. Compr Physiol.

[5] Kawai M, Rosen CJ (2010). PPARgamma: a circadian transcription factor in adipogenesis and osteogenesis. Nat Rev Endocrinol.

[6] Liu HJ, Liao HH, Yang Z, Tang QZ (2016). Peroxisome Proliferator-Activated Receptor-gamma Is Critical to Cardiac Fibrosis. PPAR Res.

[7] Reddy AT, Lakshmi SP, Reddy RC (2016). PPARgamma as a Novel Therapeutic Target in Lung Cancer. PPAR Res.

[8] Ameshima S, Golpon H, Cool CD, Chan D, Vandivier RW, Gardai SJ, Wick M, Nemenoff RA, Geraci MW, Voelkel NF (2003). Peroxisome proliferator-activated receptor gamma (PPARgamma) expression is decreased in pulmonary hypertension and affects endothelial cell growth. Circ Res.

[9] Hansmann G, de Jesus Perez VA, Alastalo TP, Alvira CM, Guignabert C, Bekker JM, Schellong S, Urashima T, Wang L, Morrell NW, Rabinovitch M (2008). An antiproliferative BMP-2/PPARgamma/apoE axis in human and murine SMCs and its role in pulmonary hypertension. J Clin Invest.

[10] Li M, Li Z, Sun X, Yang L, Fang P, Liu Y, Li W, Xu J, Lu J, Xie M, Zhang D (2010). Heme oxygenase-1/p21WAF1 mediates peroxisome proliferator-activated receptor-gamma signaling inhibition of proliferation of rat pulmonary artery smooth muscle cells. FEBS J.

[11] Kim EK, Lee JH, Oh YM, Lee YS, Lee SD (2010). Rosiglitazone attenuates hypoxia-induced pulmonary arterial hypertension in rats. Respirology.

[12] Zhang D, Wang G, Han D, Zhang Y, Xu J, Lu J, Li S, Xie X, Liu L, Dong L, Li M (2014). Activation of PPAR-gamma ameliorates pulmonary arterial hypertension via inducing heme oxygenase-1 and p21(WAF1): an in vivo study in rats. Life Sci.

[13] Tao H, Yang JJ, Shi KH, Li J (2016). Wnt signaling pathway in cardiac fibrosis: New insights and directions. Metabolism.

[14] Boonchai W, Walsh M, Cummings M, Chenevix-Trench G (2000). Expression of beta-catenin, a key mediator of the WNT signaling pathway, in basal cell carcinoma. Arch Dermatol.

[15] Qian J, Niu M, Zhai X, Zhou Q, Zhou Y (2012). β-Catenin pathway is required for TGF-β1 inhibition of PPARγ expression in cultured hepatic stellate cells. Pharmacol Res.

[16] Sabatino L (2014). Emerging role of the β-catenin-PPARγ axis in the pathogenesis of colorectal cancer. World J Gastroenterol.

[17] Lin LC, Hsu SL, Wu CL, Hsueh CM (2014). TGFβ can stimulate the p38/β-catenin/PPARγ signaling pathway to promote the EMT, invasion and migration of non-small cell lung cancer (H460 cells). Clin Exper Met.

[18] Lecarpentier Y, Vallee A (2016). Opposite Interplay between PPAR Gamma and Canonical Wnt/Beta-Catenin Pathway in Amyotrophic Lateral Sclerosis. Front Neurol.

[19] Zhu PY, Yin WH, Wang MR, Dang YY, Ye XY (2015). Andrographolide suppresses melanin synthesis through Akt/GSK3β/β-catenin signal pathway. J Dermatol Sci.

[20] Liou SF, Hsu JH, Chen YT, Chen IJ, Yeh JL (2015). KMUP-1 Attenuates Endothelin-1-Induced Cardiomyocyte Hypertrophy through Activation of Heme Oxygenase-1 and Suppression of the Akt/GSK-3β, Calcineurin/NFATc4 and RhoA/ROCK Pathways. Molecules.

[21] Hui J, Zhang J, Kim H, Tong C, Ying Q, Li Z, Mao X, Shi G, Yan J, Zhang Z, Xi G (2014). Fluoxetine Regulates Neurogenesis in vitro Through Modulation of GSK-3/−Catenin Signaling. Int J Neuropsychopharm.

[22] Pramanik KC, Fofaria NM, Gupta P, Ranjan A, Kim SH, Srivastava SK (2015). Inhibition of beta-catenin signaling suppresses pancreatic tumor growth by disrupting nuclear beta-catenin/TCF-1 complex: critical role of STAT-3. Oncotarget.

[23] Kollipara RK, Kittler R (2015). An integrated functional genomic analysis identifies the antitumorigenic mechanism of action for PPARgamma in lung cancer cells. Genom Data.

[24] Nisbet RE, Sutliff RL, Hart CM (2007). The role of peroxisome proliferator-activated receptors in pulmonary vascular disease. PPAR Res.

[25] Mansure JJ, Nassim R, Chevalier S, Szymanski K, Rocha J, Aldousari S, Kassouf W (2013). A novel mechanism of PPAR gamma induction via EGFR signalling constitutes rational for combination therapy in bladder cancer. PLoS One.

[26] Bijli KM, Kleinhenz JM, Murphy TC, Kang BY, Adesina SE, Sutliff RL, Hart CM (2015). Peroxisome proliferator-activated receptor gamma depletion stimulates Nox4 expression and human pulmonary artery smooth muscle cell proliferation. Free Radic Biol Med.

[27] Green DE, Murphy TC, Kang BY, Kleinhenz JM, Szyndralewiez C, Page P, Sutliff RL, Hart CM (2012). The Nox4 inhibitor GKT137831 attenuates hypoxia-induced pulmonary vascular cell proliferation. Am J Respir Cell Mol Biol.

[28] Wang J, Yang K, Xu L, Zhang Y, Lai N, Jiang H, Zhang Y, Zhong N, Ran P, Lu W (2013). Sildenafil inhibits hypoxia-induced transient receptor potential canonical protein expression in pulmonary arterial smooth muscle via cGMP-PKG-PPARgamma axis. Am J Respir Cell Mol Biol.

[29] Jiang Q, Lu W, Yang K, Hadadi C, Fu X, Chen Y, Yun X, Zhang J, Li M, Xu L, Tang H, Yuan JX, Wang J (2016). Sodium tanshinone IIA sulfonate inhibits hypoxia-induced enhancement of SOCE in pulmonary arterial smooth muscle cells via the PKG-PPAR-gamma signaling axis. Am J Physiol Cell Physiol.

[30] Yang K, Lu W, Jiang Q, Yun X, Zhao M, Jiang H, Wang J (2015). Peroxisome Proliferator-Activated Receptor gamma-Mediated Inhibition on Hypoxia-Triggered Store-Operated Calcium Entry. A Caveolin-1-Dependent Mechanism. Am J Respir Cell Mol Biol.

[31] Rabinovitch M (2010). PPARgamma and the pathobiology of pulmonary arterial hypertension. Adv Exp Med Biol.

[32] Green DE, Murphy TC, Kang BY, Searles CD, Hart CM (2015). PPARgamma Ligands Attenuate Hypoxia-Induced Proliferation in Human Pulmonary Artery Smooth Muscle Cells through Modulation of MicroRNA-21. PLoS One.

[33] McCubrey JA, Rakus D, Gizak A, Steelman LS, Abrams SL, Lertpiriyapong K, Fitzgerald TL, Yang LV, Montalto G, Cervello M, Libra M, Nicoletti F, Scalisi A (2016). Effects of mutations in Wnt/beta-catenin, hedgehog, Notch and PI3K pathways on GSK-3 activity-Diverse effects on cell growth, metabolism and cancer. Biochim Biophys Acta.

[34] Williams H, Slater S, George SJ (2016). Suppression of neointima formation by targeting beta -catenin/TCF pathway. Biosci Rep.

[35] Lin H, Angeli M, Chung KJ, Ejimadu C, Rosa AR, Lee T (2016). sFRP2 activates Wnt/beta-catenin signaling in cardiac fibroblasts: differential roles in cell growth, energy metabolism, and extracellular matrix remodeling. Am J Physiol Cell Physiol.

[36] Alapati D, Rong M, Chen S, Lin C, Li Y, Wu S (2013). Inhibition of LRP5/6-mediated Wnt/beta-catenin signaling by Mesd attenuates hyperoxia-induced pulmonary hypertension in neonatal rats. Pediatr Res.

[37] Takahashi J, Orcholski M, Yuan K, de Jesus Perez V, Mantei N (2016). PDGF-dependent β-catenin activation is associated with abnormal pulmonary artery smooth muscle cell proliferation in pulmonary arterial hypertension. FEBS Lett.

[38] Bonnet S, Paulin R, Sutendra G, Dromparis P, Roy M, Watson KO, Nagendran J, Haromy A, Dyck JR, Michelakis ED (2009). Dehydroepiandrosterone reverses systemic vascular remodeling through the inhibition of the Akt/GSK3-beta/NFAT axis. Circulation.

[39] Beurel E, Grieco SF, Jope RS (2015). Glycogen synthase kinase-3 (GSK3): Regulation, actions, and diseases. Pharmacol Ther.

[40] Ji XK, Xie YK, Zhong JQ, Xu QG, Zeng QQ, Wang Y, Zhang QY, Shan YF (2015). suppresses the proliferation of rat hepatic oval cells through modulating Wnt/β-catenin signaling pathway. Acta Pharmacologica Sinica.

[41] Nunes RO, Schmidt M, Dueck G, Baarsma H, Halayko AJ, Kerstjens HAM, Meurs H, Gosens R (2008). GSK-3/ β-catenin signaling axis in airway smooth muscle: role in mitogenic signaling. Am J Physiol Lung Cell Mol Physiol.

[42] Li B, Thrasher JB, Terranova P (2015). Glycogen synthase kinase-3: A potential preventive target for prostate cancer management. Urol Oncol.

[43] Penas C, Mishra JK, Wood SD, Schürer SC, Roush WR, Ayad NG (2015). GSK3 inhibitors stabilize Wee1 and reduce cerebellar granule cell progenitor proliferation. Cell Cycle.

[44] Wu Y, Liu L, Zhang Y, Wang G, Han D, Ke R, Li S, Feng W, Li M (2014). Activation of AMPK inhibits pulmonary arterial smooth muscle cells proliferation. Exp Lung Res.

